# Effects of Systematic Diet Education Combined with Multidisciplinary Nursing on Nutritional Status and Calcium and Phosphorus Metabolism in Patients with Diabetic Kidney Disease in Uremic Phase after Treatment with Alogliptin

**DOI:** 10.1155/2022/1120242

**Published:** 2022-03-15

**Authors:** Ning Guo, Na Li, Yan Zhao, Huaibin Sun, Kao Liu

**Affiliations:** Department of Organ Transplantation, Qilu Hospital of Shandong University, Jinan 250012, Shandong, China

## Abstract

**Objective:**

To explore the effects of systematic diet education combined with multidisciplinary nursing on nutritional status and calcium and phosphorus metabolism in patients with diabetic kidney disease (DKD) in uremic phase after treatment with alogliptin.

**Methods:**

A total of 90 DKD patients with uremia admitted to our hospital from January 2020 to January 2021 were selected as the research objects. The subjects were divided into combined group and routine group by random number table method. All patients received alogliptin medication. The combination group received systematic dietary education combined with multidisciplinary nursing after the medication, and the conventional group received conventional intervention. Serum albumin, blood calcium, and other indexes were detected between both groups after intervention.

**Results:**

After intervention, compared with the conventional group, all nutritional indexes of the combined group were obviously higher, levels of serum phosphorus and calcium-phosphorus product of the combined group were obviously lower (*P* < 0.001), the incidence of hypoglycemia and hyperglycemia of the combined group was obviously lower (*P* < 0.05), the total compliance rate of the combined group was obviously higher (*P* < 0.05), and the SAS score of the combined group was obviously lower (*P* < 0.001).

**Conclusion:**

With conspicuous intervention effect, systematic diet education combined with multidisciplinary nursing is a reliable method that can improve the nutritional status and levels of calcium and phosphorus metabolism, enhance treatment compliance, and reduce anxiety. Further research will help to provide a better solution for patients. This trial is registered with ChiCTR2200057011.

## 1. Introduction

Diabetic kidney disease (DKD) is one of the common complications of diabetes mellitus [1]. The monitoring of chronic diseases and their risk factors in China shows that the prevalence of diabetes in residents over 18 years old is as high as 10.4%, with the largest number of diabetic patients in China and the prevalence of DN up to 33.6% [2]. Characterized by the presence of pathological quantities of urine albumin excretion, reduced glomerular filtration rate (GFR), and increased blood pressure, DKD is considered as the main cause of end-stage renal disease (ESRD) [3]. As the end-stage manifestation of renal failure, uremia can lead to kidney failure, acid-base imbalance of water, and electrolyte and renal endocrine dysfunction, with a lot of poisoning symptoms, which seriously affects the patients' quality of life [4, 5]. Alogliptin, a highly selective oral inhibitor of the enzymatic activity of dipeptidyl peptidase-4 (DPP-4), can inhibit the activity of DPP-4 and promote the release of more endogenous glucagon-like peptide-1 to increase the number of insulin *β* cells, inhibit the aging of insulin *β* cells, and regulate blood glucose, which has been widely used in the clinical treatment [6]. According to the new guidelines for the prevention and treatment of diabetes [7], if the indexes of blood glucose are still unsatisfactory after treatment of metformin alone, DPP-4 inhibitors can be added for combined treatment. Malnutrition usually occurs in DKD patients, especially in elderly patients, which is because they have large protein consumption, poor appetite, and less intake of energy and protein than the recommended intake, resulting in poor dietary nutrition supply. Therefore, reasonable and efficient clinical interventions can be used to improve the nutritional status based on meditation treatment [8]. In recent years, systematic diet education is a new way to equip patients with systematic and all-round diet knowledge and improve their nutritional status, which has been applied in maintenance hemodialysis patients [9]. In recent years, the medical mode has gradually changed from the single biomedical one to biological, psychological, and social medical one, and multidisciplinary cooperation has been gradually used in the diagnosis and treatment of patients with DKD [10]. Multidisciplinary nursing is performed by a patient-centered nursing team which is formed by various professionals. Comprehensive and scientific nursing measures are formulated after group communication and consultation combined with patients' individual differences, so as to provide quality nursing service [11]. Multidisciplinary nursing has been applied in the treatment of patients with spinal tumor resection [12]. At present, there are few reports on the efficacy of systematic diet education combined with multidisciplinary nursing in patients with DKD in uremic phase. Therefore, the study aims to confirm the clinical application value of the combined treatment method, and the results are as follows.

## 2. Methods

### 2.1. Common Data

A total of 90 DKD patients with uremia admitted to our hospital from January 2020 to January 2021 were selected as the research objects. The subjects were divided into combined group and routine group by random number table method. This study was in line with the Declaration of Helsinki (2013) [13].

#### 2.1.1. Inclusion Criteria

It included patients who met the diagnostic criteria of DKD in uremic phase in Internal Medicine [14], patients who had good compliance, and those who did not take any medication such as vitamins or angiotensin-converting enzyme inhibitors in recent 1 month. The diagnostic criteria of DKD in uremic phase included a history of diabetes and three times of urine protein examinations in three consecutive months with the urinary excretion above 20–300 *μ*g/min while other causes of increased urinary protein excretion were excluded. The clinical symptoms included frequent urination, foamy urine, dizziness, nausea, vomiting, and edema of the lower limbs.

#### 2.1.2. Exclusion Criteria

It included patients with acute heart failure, patients who were allergic to alogliptin, patients who were pregnant or lactating, and those who were complicated with malignant tumors.

### 2.2. Treatments

All patients were treated with alogliptin. Patients orally took 25 mg/time of alogliptin (manufacturer: Japan Takeda Pharmaceutical Co., Ltd.; NMPA Approval No. H20130548; specification: 25 mg *∗* 10 s) 1 time/day for continuous 12 weeks.

(i) The conventional groups were treated with conventional nursing intervention after medication treatment, including medication guidance, exercise guidance, and self-observation.
(ii) The combined group was given systematic diet education combined with multidisciplinary nursing on the basis of medication treatment.
  1. Systematic diet education: (1) an education group was set up, which consisted of an endocrinologist, a nutritionist, a specialist nurse, and three nurses, headed by a specialist nurse. Nutritionists shall give nutritional knowledge training to team members under the guidance of Expert Consensus on Medical Nutrition Therapy of Chinese and Guidelines for Medical Nutrition Therapy of Diabetes (2013), so as to ensure that each member could master the nutrition management theory and pass the corresponding knowledge examination. (2) The systematic dietary education was conducted by the group leader on Saturday during 9 : 00–11 : 00, including the causes of DKD in uremic phase, treatment methods, healthy diet, and personal life management in the way of video, picture and text, to popularize disease-related knowledge, improve the awareness of healthy diet and life, and enhance self-management ability. After the course, the nutritionist was responsible for answering questions about nutrition management for the patients. The nutrition management team closely monitored vital signs of patients and jointly discussed and formulated the diet plan.
  2. Multidisciplinary nursing: multidisciplinary nursing team consisted of an endocrinologist in charge for diabetes treatment, 2 nurses of dialysis department in charge of comprehensive care, a nutritionist in charge of daily diet for patients, and a psychological consultant in charge of daily psychological guidance. Equipping with professional certificates, all professional medical staff carried out the medical and nursing work according to their knowledge and experience [15]. The team was headed by a nurse who was responsible for the coordination and contact among members. Regular treatment and psychological counseling were performed by the multidisciplinary team to timely solve the treatment, nursing, psychological, and other problems for patients.

### 2.3. Observation Indexes

#### 2.3.1. Nutritional Status and Levels of Calcium and Phosphorus Metabolism

5 ml of fasting venous blood of both groups was collected in the morning and centrifuged for obtaining serum samples to detect the levels of serum albumin (ALB), total protein (TP), and serum prealbumin (PA). The matching kit was used to measure the levels of blood calcium and serum phosphorus and calcium-phosphorus product was calculated, with the operation strictly following the instructions for operating procedures.

The incidence of hypoglycemia and hyperglycemia after intervention was counted in the two groups (hypoglycemia: FBG ≤3.9 mmol/L; hyperglycemia: FBG >10.0 mmol/L).

#### 2.3.2. Clinical Compliance

The Compliance Scale of Patients with Maintenance Hemodialysis for End-Stage Renal Disease [16] was used to evaluate the clinical compliance before and after intervention, including four dimensions of diet (eight items), liquid intake (six items), medication (five items), and dialysis scheme (four items), with a total of 23 items. The five-level scoring method was used, and a higher score indicated better compliance. The Cronbach *α* coefficient of the scale was 0.88, and the test-retest reliability was 0.94.

#### 2.3.3. Anxiety

The Self-Rating Anxiety Scale (SAS) [17] was used to evaluate the anxiety status before and after intervention. The scale was compiled by Zung et al. in 1971 and has been widely used to measure anxiety in general population and clinical patients. The scale included 20 items and adopted a Likert 4-level scoring method, with 1 point as “almost no or occasionally,” 2 points as “sometimes,” 3 points as “often,” and 4 points as “always.” The score of each item was added as the rough score of the scale, and the rough score multiplied by 1.25 was the standard score of the scale. A higher standard score indicated more anxiety, with a standard score ≥50 points showing positive anxiety, 50–59 showing mild anxiety, 60–69 showing moderate anxiety, and 70 and above showing severe anxiety. This scale was widely used to evaluate the anxiety of patients with good reliability and validity, and its Cronbach *α* coefficient was 0.759.

### 2.4. Statistical Analysis

All experimental data of the study were processed by SPSS23.0, and the pictures were graphed by GraphPad Prism 7 (GraphPad Software, San Diego, USA). Enumeration data was tested by *X*^2^ and expressed by [*n* (%)]. Measurement data was tested by *t* and expressed by mean ± SD. The differences were statistically significant at *P* < 0.05.

## 3. Results

### 3.1. Comparison of Clinical Data

No significant difference was found in clinical data such as sex ratio, marital status, hemoglobin, and education degree between the two groups (*P* > 0.05, see Table 1.

### 3.2. Comparison of Nutritional Indexes

After intervention, compared with the conventional group, all nutritional indexes of the combined group were obviously higher (*P* < 0.001), see Table 2.

### 3.3. Comparison of Levels of Calcium and Phosphorus Metabolism

After intervention, compared with the conventional group, levels of serum phosphorus and calcium-phosphorus product of the combined group were obviously lower (*P* < 0.001), see Table 3.

### 3.4. Comparison of Incidence of Hypoglycemia and Hyperglycemia

After intervention, compared with the conventional group, the incidence of hypoglycemia and hyperglycemia of the combined group was obviously lower (*P* < 0.05), see Figure 1.

### 3.5. Comparison of Clinical Compliance

After intervention, compared with the conventional group, the clinical compliance scores of the combined group were obviously higher (*P* < 0.05), see Table 4.

### 3.6. Comparison of Anxiety Status

No obvious difference in the SAS scores was found between the two groups before intervention (*P* > 0.05). After intervention, compared with the conventional group, the SAS score of the combined group was obviously lower (*P* < 0.001), see Table 5.

## 4. Discussion

- With the increasing incidence, DKD is far more common in the world. It is a progressive renal disease, which changes the structure and function of glomerular capillaries and renal tubules due to glucose homeostasis disorder. Studies have shown the joint effect of hemodynamic parameters, metabolism, and inflammation results in the progress of DKD [18]. DKD in uremic phase causes heart failure, myocardial infarction, and neurological disorders such as uremic encephalopathy and convulsions. As a common microvascular complication of diabetes, DKD is mainly characterized by urinary microalbuminosis in the early stage, which is reversible. If poorly controlled, it can seriously damage the renal function of patients at the stage of massive proteinuria, eventually leading to uremia [19]. As a highly selective DPP-4 inhibitor, alogliptin can increase the levels of glucose-dependent insulinotropic peptide and glucagon-like peptide-1, promote the differentiation and proliferation of pancreatic *β* cell, inhibit pancreatic *α* cell, reduce the excessive secretion of glucagon, and control the blood glucose level [20, 21]. However, clinical practice has proved that medication treatment alone cannot achieve conspicuous curative effect. Diet education, an economic and effective method for the treatment of DKD, can significantly promote the control and management of DKD and regulate blood glucose, blood pressure, and blood lipid levels of patients. Some scholars put forward that exercise combined with diet education can improve blood sugar, blood fat, and 25-hydroxy vitamin D levels in patients with DKD [22], which provides a new idea for the treatment of DKD in uremic phase.
- The investigation shows that due to ignorance of their own diseases and poor clinical compliance, patients with DKD in uremic phase have poor blood glucose control and rapid progress, which may lead to readmission in a short time. Therefore, the implementation of efficient clinical management measures is of great significance to control the progress of the disease and improve the prognosis [23]. In this study, with the help of relevant literature and previous clinical experience, the systematic diet education combined with multidisciplinary nursing on the basis of alogliptin treatment was used in patients with DKD in uremic phase. By comparing the compliance and anxiety status of the two groups after treatment, the clinical compliance of the combined group was remarkably higher than those of the conventional group, and SAS score of the combined group was remarkably lower than those of the conventional group (*P* < 0.05). It is speculated that the systematic diet education enables the patients to master the disease-related knowledge through training and greatly enhance self-management ability, which has been confirmed in patients with non-Hodgkin lymphoma [24]. Moreover, multidisciplinary nursing equips with professional nursing staff and psychological consultant, which can better provide quality service as well as relieve pressure for patients.
- With the longer course of DKD, persistent hyperglycemia, insulin resistance, and obesity will lead to osteoporosis. In addition, increased dialysis of glomerular filtration membrane and disorder of calcium and phosphorus metabolism will cause secondary parathyroid hyperfunction and damage the sclerotin [25]. The results of this study confirmed that patients in the combined group had significantly better nutritional status after intervention than those in the conventional group (*P* < 0.001), indicating that the clinical combined nursing intervention could improve the malnutrition and strengthen physical fitness for patients.

### 4.1. Limitations of the Study

This study is limited by the small sample size and the single sample source, which is lack of representativeness. Meanwhile, the study time is short, without long-term follow-up observation, so the efficacy of the combined intervention cannot be evaluated accurately. Therefore, it is necessary to further improve the treatment method, prolong the follow-up time, and expand the sample size by carrying out multicenter research.

## 5. Conclusion

With conspicuous treatment effect, systematic diet education combined with multidisciplinary nursing can improve the nutritional status and levels of calcium and phosphorus metabolism, enhance treatment compliance, and reduce anxiety, which should be applied into the clinical nursing.

## Figures and Tables

**Figure 1:** Comparison of incidence of hypoglycemia and hyperglycemia [*n* (%)]. (a) The comparison of incidence of hypoglycemia between the two groups after intervention. The abscissa indicates the combined group and the conventional group, and the ordinate indicates cases of hypoglycemia. The incidence of hypoglycemia in the combined group and the conventional group after intervention was 2 cases (4.44%) and 9 cases (20.00%), respectively. ^*∗*^indicates the obvious difference in incidence of hypoglycemia between the two groups after intervention (*X*^2^ = 5.075, *P* < 0.05). (b) The comparison of incidence of hyperglycemia between the two groups after intervention. The abscissa indicates the combined group and the conventional group, and the ordinate indicates cases of hyperglycemia. The incidence of hyperglycemia in the combined group and the conventional group after intervention was 1 case (2.22%) and 7 cases (16.67%), respectively. ^*∗∗*^indicates the obvious difference in incidence of hyperglycemia between the two groups after intervention (*X*^2^ = 4.939, *P* < 0.05).

**Table 1:** Comparison of clinical data (*n* = 45).

Items	Combined group	Conventional group	*χ* ^2^/*t*/*Z*	*P*
Gender			0.182	0.670
Male	25	27		
Female	20	18		
Family monthly income (Yuan)			0.809	0.368
<3000	8	5		
≥3000	37	40		
Smoking			0.185	0.667
Yes	19	17		
No	26	28		
Drinking			0.180	0.671
Yes	21	19		
No	24	26		
Marital status			0.137	0.711
Married	40	42		
Unmarried	5	3		
Education level			0.400	0.527
Primary school and below	21	24		
Junior high school and above	24	21		
Residence			0.178	0.673
Urban area	21	23		
Rural area	24	22		
Age (years old)	59.89 ± 10.53	60.91 ± 9.33	−0.487	0.627
Course of disease	6.24 ± 3.04	6.41 ± 2.87	−0.268	0.790
BMI	20.70 ± 3.16	21.14 ± 2.54	−0.725	0.470
Fasting blood glucose	7.26 ± 1.19	7.32 ± 1.35	−0.232	0.817
Hemoglobin	90.87 ± 11.02	91.60 ± 10.18	−0.328	0.744
Total cholesterol	5.53 ± 3.18	5.49 ± 2.61	0.069	0.945

**Table 2:** Comparison of nutritional indexes (mean ± SD).

Group	Serum albumin (ALB) (g/L)	Total protein (TP) (g/L)	Serum prealbumin (PA) (mg/L)
Combined group	41.56 ± 6.97	63.12 ± 11.72	29.48 ± 5.29
Conventional group	34.57 ± 9.02	50.04 ± 12.73	23.99 ± 7.09
*t*	4.114	5.072	4.163
*P*	<0.001	<0.001	<0.001

**Table 3:** Comparison of indexes of calcium and phosphorus metabolism (mean ± SD).

Group	Serum phosphorus (mmol/L)	Blood calcium (mmol/L)	Calcium-phosphorus product (mol^2^/L)
Combined group	1.60 ± 0.65	2.51 ± 0.28	3.97 ± 1.57
Conventional group	2.94 ± 0.92	2.01 ± 0.18	5.87 ± 1.87
*t*	−6.050	−7.814	−5.197
*P*	<0.001	<0.001	<0.001

**Table 4:** Comparison of clinical compliance [*n* (%)].

Group	Diet compliance	Liquid intake compliance	Medication compliance	Compliance of dialysis scheme	Total score of treatment compliance
Combined group	31.87 ± 5.10	25.13 ± 4.36	24.16 ± 1.26	19.58 ± 0.49	100.73 ± 7.65
Conventional group	28.62 ± 6.19	22.67 ± 5.87	22.76 ± 2.49	17.44 ± 2.76	91.49 ± 13.36
*t*	2.712	−2.053	−3.271	−5.020	−3.501
*P*	0.008	0.040	0.001	<0.001	<0.001

**Table 5:** Comparison of the SAS scores between the two groups after intervention (mean ± SD).

Group	*n*	Before intervention	After intervention
Combined group	45	54.71 ± 11.20	39.09 ± 7.77
Conventional group	45	54.98 ± 12.65	50.16 ± 14.06
*t*		−0.106	−3.875
*P*		0.916	<0.001

## Data Availability

The data that support the findings of this study are available on reasonable request from the corresponding author.
